The article "Variable copy number of mitochondrial DNA (mtDNA) predicts worse prognosis in advanced gastric cancer patients" was published in 2013. Journal: Diagn Pathol.

# Variable copy number of mitochondrial DNA (mtDNA) predicts worse prognosis in advanced gastric cancer patients

**DOI:** 10.1186/1746-1596-8-173

**Published:** 2013-10-21

**Authors:** Guanjun Zhang, Yiping Qu, Siwen Dang, Qi Yang, Bingyin Shi, Peng Hou

**Affiliations:** 1 Department of Pathology, The First Affiliated Hospital of Xi’an Jiaotong University School of Medicine, Xi’an 710061, the People’s Republic of China; 2 Department of Endocrinology, The First Affiliated Hospital of Xi’an Jiaotong University School of Medicine, Xi’an 710061, the People’s Republic of China

**Keywords:** Gastric cancer, Mitochondrial DNA (mtDNA), Copy number, Real-time quantitative PCR, Clinical outcomes

## Abstract

**Background:**

Change of mitochondrial DNA (mtDNA) copy number is widely reported in various human cancers, including gastric cancer, and is considered to be an important hallmark of cancers. However, there is remarkably little consensus on the value of variable mtDNA content in the prognostic evaluation of this cancer.

**Methods:**

Using real-time quantitative PCR approach, we examined mtDNA copy number in a cohort of gastric cancers and normal gastric tissues, and explored the association of variable mtDNA content with clinical outcomes of gastric cancer patients.

**Results:**

Our data showed that the majority of gastric cancer patients had low mtDNA content as compared to control subjects although the relative mean mtDNA content was higher in the former than the latter. Moreover, we found that variable mtDNA content was strongly associated with lymph node metastasis and cancer-related death of the patients with late-stage tumors. Notably, variable mtDNA content did not affect overall survival of gastric cancer patients, however, we found that increased mtDNA content was associated with poor survival in the patients with late-stage tumors.

**Conclusion:**

In this study, we demonstrated that variable mtDNA content markedly increased the risk of lymph node metastasis and high mortality of the patients with late-stage tumors. Additionally, we found a strong link between increased mtDNA content and worse survival of the patients with late-stage tumors. Taken together, variable mtDNA content may be a valuable poor prognostic factor for advanced gastric cancer patients.

**Virtual slides:**

The virtual slide(s) for this article can be found here: http://www.diagnosticpathology.diagnomx.eu/vs/1344721463103353.

## Background

Gastric cancer is the second cause of cancer deaths after lung cancer, and is a major health burden worldwide [1]. Despite advances in therapeutic modalities during the past decades, the prognosis at the advanced stage is still dismal, with an average 5-year survival rate of less than 20% [2,3]. The cause of gastric cancer is multifactorial, and the prognosis varies widely in gastric cancer patients due to yet undetermined biologic factors [4]. Thus, there is increasing need to develop reliable biomarkers for predicting clinical outcomes and establishing new therapeutic and preventive strategies to this disease.

The article "Variable copy number of mitochondrial DNA (mtDNA) predicts worse prognosis in advanced gastric cancer patients" was published in 2013. Journal: Diagn Pathol.

Although a number of biomarkers have been demonstrated to be closely associated with poor prognosis of gastric cancer patients [5-9], most of them are concerned with the roles of nuclear DNA (nDNA) alterations in gastric tumorigenesis [10-14]. These genetic or epigenetic alterations cause gain-of-function in oncogenes and loss-of-function in tumor suppressor genes [15,16], however, relatively less attention has been paid to mitochondrial DNA (mtDNA) alterations. Mitochondria are organelles found in all nucleated cells. The major role of mitochondria is to generate cellular adenosine triphosphate (ATP) through oxidative phosphorylation [17]. Human mtDNA is a 16,569 base-pair, double-stranded, closed-circular DNA molecule that encodes 13 polypeptides, 2 rRNAs, and a set of 22 tRNAs required for protein synthesis in mitochondria [18]. The displacement loop (D-loop) is a noncoding region essential for the replication and transcription of mtDNA. Mutations in the D-loop may cause a reduction in mtDNA copy number or altered mtDNA gene expression [19,20]. Generally, each human cell contains several hundred to 1000 mitochondria, and each mitochondrion has 2 to 10 copies of mtDNA. The mitochondrial genome is more vulnerable to oxidative damage and undergoes a higher rate of mutation than does the nDNA [21,22]. Increasing evidences have demonstrated the association of increased mtDNA content in peripheral blood with increased risk of non-Hodgkin lymphoma [22], lung cancer [23], pancreatic cancer [24], breast cancer [25], and colorectal cancer [26], whereas increased risk of renal cancer is associated with decreased mtDNA content [27]. Although several studies have reported depletion in mtDNA copy number in gastric cancers as compared with normal gastric tissues [28,29], there is no relationship between leukocyte mtDNA content and the risk of developing gastric cancer [30]. Until now, the association of mtDNA content with clinical outcomes of gastric cancer patients remains largely unknown.

In the present study, we investigated mtDNA copy number in a cohort of gastric cancers and normal gastric tissues using real-time quantitative PCR approach, and explored the effect of mtDNA content on clinical outcomes of gastric cancer patients.

## Methods

### Patients

With the approval of our institutional review board and human ethics committee, where required, a total of 103 paraffin-embedded gastric cancer tissues were randomly obtained at the First Affiliated Hospital of Xi’an Jiaotong University School of Medicine between January 2000 and December 2009. A total of 33 gastric tissues from the patients with chronic gastritis who underwent endoscopic biopsy were used as control subjects. None of these patients received chemotherapy and radiotherapy before the surgery. All samples were histologically examined by a senior pathologist at Department of Pathology of the Hospital based on World Health Organization (WHO) criteria. Clinicopathological data were obtained from the patients’ files or by interview with the patients or their relatives, and were summarized in Table 1.

The article "Variable copy number of mitochondrial DNA (mtDNA) predicts worse prognosis in advanced gastric cancer patients" was published in 2013. Journal: Diagn Pathol.

**Table 1:** Clinicopathological characteristics of gastric cancer patients

**Characteristics**	**No. of patients (%)**
Gender	
Male	84 (81.5)
Female	19 (18.5)
Age, years	
Mean	58.8
SD	12.9
Tumor localization	
gastric cardia	20 (19.4)
gastric body	32 (31.1)
gastric antrum	51 (49.5)
Tumor size (cm3)	
≤3	32 (31.1)
3-5	36 (35.0)
>5	35 (33.9)
Differentiation	
well/moderate	48 (46.6)
poor/undifferentiation	55 (53.4)
Tumor invasion	
T1	23 (22.3)
T2	14 (13.6)
T3	52 (50.5)
T4	14 (13.6)
TNM stage	
I	9 (8.7)
II	41 (39.8)
III	47 (45.6)
IV	6 (5.8)
Lymph node metastasis (LNM)	
Yes	48 (46.6)
No	55 (53.4)
No. of LNM	
N0	55 (53.4)
N1 (1–6)	34 (33.0)
N2 (7–15)	10 (9.7)
N3 (≥16)	4 (3.9)
Survival status	
Dead	45 (43.7)
Alive	58 (56.3)

### DNA preparation

Serial sections from each tumor sample were cut. One section was stained using hematoxylin and eosin (H&E) and was marked as a tumor representative tissue by an expert surgical pathologist for gastric cancer. Tumor tissues were then isolated by manual microdissection under an inverted microscope using the marked H&E section for target tissue identification. DNA was extracted from isolated tumor tissues as previously described [13]. Briefly, the tissues were first treated with xylene for 12 h at room temperature to remove the paraffin, and were then subjected to digestion with 1% sodium dodecylsulfate (SDS) and proteinase K at 48°C for 48 to 72 h with addition of several spiking aliquots of concentrated proteinase K to facilitate digestion. Genomic DNA was isolated from the digested tissues followed by standard phenol-chloroform extraction and ethanol precipitation protocol, and stored at −80°C until use.

### mtDNA copy number analysis

Relative mtDNA copy number was measured in a cohot of gastric cancers and normal gastric tissues by real-time quantitative PCR method. Specific primers and TaqMan probes were designed using Primer Express 3.0 (Applied Biosystems, Foster City, CA) to amplify *MT-ND1* gene in mtDNA and the internal reference gene *β-actin*. TaqMan probes were labeled with 5′-FAM (6-carboxyfluorescein, fluorescent reporter) and 3′-TAMRA (6-carboxy-tetramethylrhodamine, fluorescent quencher). The primer and probe sequences for *MT-ND1* and *β-actin* genes were presented in Table 2. Using a PCR protocol described previously [31], PCR amplification was carried out in the buffer containing 16.6 mM ammonium sulfate, 67 mM Tris base, 2.5 mM MgCl_2_, 10 mM 2-mercaptoethanol, 0.1% DMSO, 0.2 mM each of dATP, dCTP, dGTP and dTTP, 600 nM each of forward and reverse primers, 200 nM TaqMan probe, 0.6 unit Platinum Taq polymerase and 2% Rox reference dye. Each sample was run in triplicate, and *β-actin* was run in parallel to standardize the input DNA. Standard curves were established using serial dilutions of normal leukocyte DNA with a quantity range of 6.25 to 100 ng per 2 μL. The relative mtDNA copy number of each sample was calculated as described previously [27,30].

The article "Variable copy number of mitochondrial DNA (mtDNA) predicts worse prognosis in advanced gastric cancer patients" was published in 2013. Journal: Diagn Pathol.

**Table 2:** The primer and TaqMan probe sequences used in this study

**Genes**	**Forward primer sequence (5′→3′)**	**Probe sequence (5′→3′)**	**Reverse primer sequence (5′→3′)**	**Amplification efficiency (%)**
*MT-ND1*	CCCCTAAAACCCGCCACATC	6FAM-ACCCTCTACATCACCGCCCCGACC-TAMRA	GTAGAAGAGCGATGGTGAGAGC	93.6
*β-actin*	TCACCCACACTGTGCCCATCTACGA	6FAM-ATGCCCTCCCCCATGCCATCC-TAMRA	TCGGTGAGGATCTTCATGAGGTA	95.7

### Statistical analysis

The Mann–Whitney *U* test was used to compare mtDNA copy number between gastric cancer and normal gastric tissues. Association of mtDNA copy number with clinicopathological characteristics was assessed univariately using the SPSS statistical package (version 11.5, Chicago, IL). Multivariate models were then developed that adjusted for the most important covariates, including age, tumor size, differentiation, and lymph node metastasis. Survival length was determined from the day of primary tumor surgery to the day of death or last clinical follow-up. The Kaplan–Meier method was used for survival analysis grouping with copy number variations of mtDNA. Differences between curves were analyzed using the log-rank test. Multivariate Cox regression analysis was used to evaluate the effect of mtDNA copy number on survival of independently of the number of lymph node metastasis, tumor invasion and differentiation. All statistical analyses were performed using the SPSS statistical package (version 11.5, Chicago, IL). *P* values < 0.05 were considered significant.

## Results

### Relative mtDNA copy number in gastric cancer

Real-time quantitative PCR assay was performed to analyze mtDNA copy number in 103 gastric cancers and 33 normal gastric tissues. As shown in Figure 1, the relative mean mtDNA content was higher in gastric cancer patients (6.06 ± 8.76 copies) than control subjects (4.48 ± 2.46 copies). However, the difference did not reach statistical significance (*P* =0.171). The median values among gastric cancer patients and control subjects were 2.94 copies (range = 0.39-50.12 copies) and 4.07 copies (range = 0.34-10.10 copies), respectively, suggesting that the majority of gastric cancer patients had low mtDNA content as compared to control subjects, as supported by the previous studies [28,29]. We next evaluated whether mtDNA content differed by selected clinicopathological characteristics. As shown in Figure 2, overall, we did not find significant differences in mtDNA copies by gender, age, tumor localization, tumor size, differentiation, tumor invasion, TNM stage, lymph node metastasis and survival status. Notably, although no statistical significance was noted, the patients with lymph node metastasis had a lower mtDNA content than the patients without lymph node metastasis (4.45 *vs.* 7.46 copies, *P* =0.12) (Figure 2). Moreover, mtDNA content in gastric antrum was lower than that in gastric cardia and body (4.66 *vs.* 6.51 and 7.99 copies) (Figure 2).

The article "Variable copy number of mitochondrial DNA (mtDNA) predicts worse prognosis in advanced gastric cancer patients" was published in 2013. Journal: Diagn Pathol.

**Figure 1:** **Copy number of mtDNA corresponding to each individual case of gastric cancers and normal gastric tissues (circle).** Real-time quantitative PCR assay was performed to analyze mtDNA copy number in a cohort of gastric cancers and normal gastric tissues. Horizonal lines represent mean ± S.E. Details are as described in Methods. T, tumor tissues; N, normal gastric tissues.

**Figure 2:** **Association of mtDNA copy number with clinicopathological characteristics in gastric cancer.** Copy number of mtDNA was analyzed using real-time quantitative PCR approach. The circle represents mtDNA copy number of each case of gastric cancers. Horizonal lines represent mean ± S.E. Sample means were compared using the Mann–Whitney *U* test. Details are as described in Methods. F, female; M, male; GC, gastric cardia; GA, gastric antrum; GB, gastric body; Well, well/moderate differentiation; Poor, poor/undifferentiation; N, non-lymph node metastasis; Y, lymph node metastasis; ES, early-stage; LS, late-stage.

### Association of variable mtDNA content with clinicopathological characteristics of gastric cancer patients

To further examine the relationship of mtDNA content with clinicopathological characteristics of gastric cancer patients, we chosed two cutoff points, which are the lower and upper limit (3.61 and 5.35 copies) of the overall 95% confidence interval for all control subjects, respectively. Gastric cancer patients were then categorized into three groups by use of these two cutoff points, including individuals with highest (>5.35 copies) (termed “increased mtDNA content” hereafter), medium (3.61-5.35 copies) and lowest (<3.61 copies) (termed “decreased mtDNA content” hereafter) category of mtDNA content. Medium category of mtDNA content (3.61-5.35 copies) was used as a reference. As shown in Table 3, variable mtDNA content was closely associated with lymph node metastasis in gastric cancer patients. Compared with the reference, decreased mtDNA content significantly increased the risk of lymph node metastasis in gastric cancer patients (OR =4.93, 95% CI =1.28-19.04, *P* =0.02). Similarly, although the association did not reach statistical difference, increased mtDNA content also increased the risk of lymph node metastasis of patients (OR =4.00, 95% CI =0.91-17.58, *P* =0.07).

The article "Variable copy number of mitochondrial DNA (mtDNA) predicts worse prognosis in advanced gastric cancer patients" was published in 2013. Journal: Diagn Pathol.

**Table 3:** Copy number variations of mtDNA in gastric cancer — univariate associations with clinicopathological characteristics

**Characteristics**	** Copy number <3.61**		** Copy number >5.35**	
	OR^* ^**(95% CI)**	***P***	OR^* ^**(95% CI)**	***P***
Male *vs.* Female	1.55 (0.42-5.70)	0.51	1.75 (0.37-8.30)	0.48
Age^1^	1.00 (0.65-1.52)	0.98	1.10 (0.67-1.79)	0.71
Tumor localization^2^	1.11 (0.51-2.42)	0.80	1.22 (0.50-2.99)	0.66
Tumor size^3^	1.31 (0.66-2.60)	0.45	1.37 (0.63-3.01)	0.43
Differentiation^4^	1.78 (0.58-5.49)	0.32	1.11 (0.31-4.04)	0.87
Tumor invasion^5^	0.82 (0.46-1.47)	0.50	0.69 (0.36-1.34)	0.27
TNM stage^6^	0.84 (0.40-1.78)	0.65	0.86 (0.36-2.03)	0.73
Lymph node metastasis	4.93 (1.28-19.04)	0.02	4.00 (0.91-17.58)	0.07
Survival status^7^	1.20 (0.39-3.73)	0.75	1.81 (0.50-6.50)	0.37

*OR: odds ratio with 95% confidence interval; ^1^Age (per 10 years); ^2^Tumor localization (gastric cardia; gastric body; gastric antrum); ^3^Tumor size (≤3 cm; >3 cm and ≤5 cm; >5 cm); ^4^Differentiation (well or moderate; poor or undifferentiation); ^5^Tumor invasion (T1; T2; T3; T4); ^6^TNM stage (I; II; III; IV); ^7^Survival status (Alive *vs.* Dead). The cases with 3.61-5.35 mtDNA copies were used as reference.

Gastric cancer patients were further categorized into two groups based on TNM stage, such as individuals with early-stage (stages I and II) and late-stage (stages III and IV) tumors. As shown in Table 4, increased mtDNA content was significantly negatively associated with tumor invasion in the patients with early-stage tumors (OR =0.28, 95% CI =0.08-0.99, *P* =0.049). Both decreased and increased mtDNA content dramatically increased the risk of lymph node metastasis for the patients with late-stage tumors (the former: OR =27.00, 95% CI =2.89-252.62, *P* =0.004; the latter: OR =13.50, 95% CI =1.34-135.98, *P* =0.03) (Table 5). Also shown in Table 5, increased mtDNA content was significantly associated with higher mortality of the patients with late-stage tumors (OR =6.42, 95% CI =1.09-37.74, *P* =0.04) (Table 5). Moreover, decreased mtDNA also increased the risk of caner-related death in advanced gastric cancer patients (OR =3.11, 95% CI =0.66-14.60, *P* =0.15), although no statistical significance was found. In order to assess the independent association of variable mtDNA content with age, tumor size, differentiation and lymph node metastasis, we conducted a multivariable logistic regression. As shown in Table 6, similar to univariate analysis, both decreased and increased mtDNA content remained closely associated with lymph node meatstasis after adjustment, particularly the former (OR =7.63, 95% CI =1.63-35.69, *P* =0.01). Moreover, although we did not find statistical significance, deceased mtDNA content was positively associated with poor differentiation of gastric cancer patients (OR =3.00, 95% CI =0.86-10.47, *P* =0.08) (Table 6).

The article "Variable copy number of mitochondrial DNA (mtDNA) predicts worse prognosis in advanced gastric cancer patients" was published in 2013. Journal: Diagn Pathol.

**Table 4:** Copy number variations of mtDNA in early-stage gastric cancer — univariate associations with clinicopathological characteristics

**Characteristics**	** Copy number <3.61**		** Copy number >5.35**	
	OR^* ^**(95% CI)**	***P***	OR^* ^**(95% CI)**	***P***
Male *vs.* Female	1.16 (0.11-12.13)	0.90	0.80 (0.06-11.30)	0.87
Age^1^	0.48 (0.05-4.65)	0.53	0.20 (0.02-2.39)	0.20
Tumor localization^2^	3.65 (0.91-14.64)	0.07	2.78 (0.59-13.0)	0.19
Tumor size^3^	0.80 (0.24-2.65)	0.71	0.56 (0.13-2.32)	0.42
Tumor invasion^4^	0.49 (0.16-1.49)	0.21	0.28 (0.08-0.99)	0.049
Lymph node metastasis	1.09 (0.17-6.85)	0.93	0.86 (0.10-7.51)	0.90
Survival status^5^	0.42 (0.07-2.43)	0.33	0.25 (0.03-2.32)	0.22

*OR: odds ratio with 95% confidence interval; ^1^Age (per 10 years); ^2^Tumor localization (gastric cardia; gastric body; gastric antrum); ^3^Tumor size (≤3 cm; >3 cm and ≤5 cm; >5 cm); ^4^Tumor invasion (T1; T2; T3; T4); ^5^Survival status (Alive *vs.* Dead). The cases with 3.61-5.35 mtDNA copies were used as reference.

**Table 5:** Copy number variations of mtDNA in late-stage gastric cancer — univariate associations with clinicopathological characteristics

**Characteristics**	** Copy number <3.61**		** Copy number >5.35**	
	OR^* ^**(95% CI)**	***P***	OR^* ^**(95% CI)**	***P***
Male *vs.* Female	1.57 (0.31-7.99)	0.59	2.79 (0.37-20.82)	0.32
Age^1^	0.67 (0.15-2.89)	0.59	1.33 (0.25-7.01)	0.73
Tumor localization^2^	0.44 (0.13-1.45)	0.18	0.70 (0.19-2.616)	0.60
Tumor size^3^	1.86 (0.78-4.42)	0.16	2.10 (0.79-5.57)	0.14
Tumor invasion^4^	1.13 (0.53-2.41)	0.74	1.16 (0.50-2.69)	0.73
Lymph node metastasis	27.00 (2.89-252.62)	0.004	13.50 (1.34-135.98)	0.03
Survival status^5^	3.11 (0.66-14.60)	0.15	6.42 (1.09-37.74)	0.04

*OR: odds ratio with 95% confidence interval; ^1^Age (per 10 years); ^2^Tumor localization (gastric cardia; gastric body; gastric antrum); ^3^Tumor size (≤3 cm; >3 cm and ≤5 cm; >5 cm); ^4^Tumor invasion (T1; T2; T3; T4); ^5^Survival status (Alive *vs.* Dead). The cases with 3.61-5.35 mtDNA copies were used as reference.

The article "Variable copy number of mitochondrial DNA (mtDNA) predicts worse prognosis in advanced gastric cancer patients" was published in 2013. Journal: Diagn Pathol.

**Table 6:** Copy number variations in gastric cancer — multivariable models assessing age, tumor size, differentiation and lymph node metastasis

**Characteristics**	** Copy number <3.61**		** Copy number >5.35**	
	OR^* ^**(95% CI)**	***P***	OR^* ^**(95% CI)**	***P***
Age^1^	0.80 (0.49-1.31)	0.38	0.96 (0.56-1.65)	0.89
Tumor size^2^	0.91 (0.43-1.92)	0.80	1.04 (0.46-2.36)	0.92
Differentiation^3^	3.00 (0.86-10.47)	0.08	1.56 (0.39-6.19)	0.53
Lymph node metastasis	7.63 (1.63-35.69)	0.01	4.41 (0.84-23.12)	0.08

*OR: odds ratio with 95% confidence interval; ^1^Age (per 10 years); ^2^Tumor size (≤3 cm; >3 cm and ≤5 cm; >5 cm); ^3^Differentiation (well or moderate; poor or undifferentiation). The cases with 3.61-5.35 mtDNA copies were used as reference.

### Effect of variable mtDNA content on poor survival of gastric cancer patients

Given that variable mtDNA content is associated with some of clinicopathological features in gastric cancer patients, we next investigated its association with poor survival. Similarly, medium category of mtDNA content (3.61-5.35 copies) was used as a reference in this study. As shown in Table 7, variable mtDNA content did not affect overall survival of gastric cancer patients. We then used Kaplan-Meier survival curves to further determine the effect of variable mtDNA content on the survival of gastric cancer patients. Similar to the findings in Table 7, decreased or increased mtDNA content did not significantly affect survival time of gastric cancer patients (the former: 54.2 months *vs.* 51.4 months on average, *P* =0.93; the latter: 44.4 months *vs.* 51.4 months on average, *P* =0.38) (Figure 3). Cox multivariate repression showed that decreased or increased mtDNA content (the former: HR =0.52, 95% CI =0.20-1.38, *P* =0.19; the latter: HR =1.07, 95% CI =0.37-3.07, *P* =0.90*)* is not a predictor of poor survival for gastric cancer patients as an independently variable with respect to the number of lymph node metastasis, tumor invasion and differentiation. The data were stratified further based on the TNM tumor stage, because it is an independent risk factor for gastric cancer patients. Also shown in Figure 3, decreased or increased mtDNA content did not affect survival time of the patients with early-stage tumors (the former: 60.6 months *vs.* 55.3 months on average, *P =*0.24; the latter: 61.2 months *vs.* 55.3 months on average, *P =*0.25). However, increased mtDNA content was markedly associated with poor survival of the patients with late-stage tumors as compared with the reference (33.1 months *vs.* 49.3 months on average, *P =*0.05) (Figure 3).

The article "Variable copy number of mitochondrial DNA (mtDNA) predicts worse prognosis in advanced gastric cancer patients" was published in 2013. Journal: Diagn Pathol.

**Table 7:** Prognostic value of clinicopathological factors and copy number variation of mtDNA in univariate and multivariate Cox regression analysis (n=103)

	**Univariate analysis**		**Multivariate analysis**	
**Variable**	**Hazard ratio (95% CI)**	***P***	**Hazard ratio (95% CI)**	***P***
Copy number				
3.61~5.35	1.00 (reference)		1.00 (reference)	
<3.61	1.51 (0.44-2.57)	0.90	0.52 (0.20-1.38)	0.19
>5.35	1.53 (0.58-4.02)	0.39	1.07 (0.37-3.07)	0.90
The number of lymph node metastasis				
0	1.00 (reference)		1.00 (reference)	
1~6	6.86 (3.18-14.91)	<0.001	7.28 (2.87-18.49)	<0.001
7~15	6.41 (2.70-15.25)	<0.001	4.68 (1.65-13.28)	0.004
≥16	16.75 (5.05-55.56)	<0.001	13.21 (3.33-52.45)	<0.001
Tumor invasion				
T1	1.00 (reference)		1.00 (reference)	
T2	0.85 (0.16-4.67)	0.86	0.63 (0.11-3.54)	0.60
T3	4.36 (1.53-12.42)	0.006	1.51 (0.46-4.92)	0.49
T4	2.66 (1.30-5.48)	0.001	3.33 (0.92-12.14)	0.07
Differentiation				
Well/moderate	1.00 (reference)		1.00 (reference)	
Poor/undifferentiation	2.22 (1.19-4.19)	0.01	1.82 (0.86-3.82)	0.12

**Figure 3:** **The effect of variable mtDNA content on poor survival of gastric cancer patients.** Kaplan-Meier analysis of survival was performed according to copy number variations of mtDNA in a large cohort of gastric cancers. Kaplan-Meier survival curves show that variable (decreased or increased) mtDNA content was not associated with overall survival of the patients. However, when the data were stratified further based on the TNM tumor stage, increased mtDNA content (>5.35 copies) was strongly associated with worse survival in the patients who had late-stage tumors.

## Discussion

Although much of the current funding is aligned to continuing to further understand the functional details of the nuclear genome, the mitochondrion and its modest complement of DNA and protein is emerging as a crucial component of the biological networking of nuclear pathways [18]. Mitochondria are eukaryotic organelles involved in many important physiological processes, including metabolism, signaling, apoptosis, cell cycle, differentiation and responsible for energy production [32]. It has been well documented that the enhanced production of mitochondrial reactive oxygen species (ROS), most notably superoxide, hydroxyl radicals, and hydrogen peroxide is a prominent byproduct of cancer cell metabolism [33]. Within various cells, tissues and organs, mtDNA copy number is different, and this difference can also occur in a given type of cell under different conditions or internal or external microenvironments [34,35]. Unlike nuclear DNA, mtDNA is present at a consistently high level in each cell [36], and mtDNA mutation rate is much higher than that of nuclear DNA [18,21]. Mitochondrial aberrants, including mtDNA mutations and copy number variations, have been frequently identified in different types of human cancers, including gastric cancer [28-30,36,37], suggesting that mtDNA aberrations play a critical role in gastric tumorigenesis. However, the prognostic values of mtDNA aberrants, particularly copy number variations, in gastric cancer patients ramain largely unclear.

The article "Variable copy number of mitochondrial DNA (mtDNA) predicts worse prognosis in advanced gastric cancer patients" was published in 2013. Journal: Diagn Pathol.

In this study, we investigated relative mtDNA copy number in a cohort of gastric cancers and normal gastric tissues (control subjects) using real-time quantitative PCR approach. Our data showed that the majority of the cancer patients had low levels of mtDNA copy number as compared to control subjects, although mean mtDNA content was a little bit higher in gastric cancer patients than control subjects. In line with this study, the previous studies have demonstrated that mtDNA depletion is frequently found in gastric cancers as compared with normal gastric tissues [28,29], implicating that low mtDNA content is involved in the formation and progression of gastric cancer. Moreover, we did not find the association of mtDNA content with most of clinicopathological features, such as gender, age, tumor localization, tumor size, differentiation, tumor invasion, TNM stage and survival status. However, we found that the patients with lymph node metastasis had a lower mtDNA copy number than the patients without lymph node metastasis, although the difference between two groups was not statistically significant.

To further explore the association of mtDNA content with clinicopathological characteristics and poor survival of gastric cancer patients, we categorized the patients into three groups based on two cutoff points (the lower and upper limit of 95% confidence interval for all control subjects), such as decreased mtDNA content (<3.61 copies), normal mtDNA content or reference (3.61-5.35 copies) and increased mtDNA content (>5.35 copies). Our findings showed that variable mtDNA content (whatever decreased or increased mtDNA content) was closely associated with an increased risk of lymph node metastasis for gastric cancer patients as compared to reference. Strikingly, when gastric cancer patients were further categorized into early-stage and late-stage groups based on TNM stage, variable mtDNA content was not asscoiated with lymph node metastasis for the patients with early-stage tumors. However, both decreased and increased mtDNA content significantly increased the risk of of lymph node metastasis for the patients with late-stage tumors. These observations suggest that copy number variations of mtDNA may be invloved in gastric cancer progression. Similar to our findings in the present study, a previous study showed that mtDNA content was increased gradually from the non-cancerous esophageal mucosa to esophageal squamous cell carcinoma (ESCC) and then the metastatic lymph nodes [38]. Moreover, our data showed that variable mtDNA content was associated with cancer-related death of the patients with late-stage tumors. Collectively, our findings suggest that variable mtDNA content may contribute to poor clinical outcomes of gastric cancer patients, particularly the patients with advanced tumors. Next, we evaluated the effect of variable mtDNA content on poor survival of gastric cancer patients. Our data showed that both decreased and increased mtDNA content were not associated with overall survival of gastric cancer patients. However, when the patients were categorized into early-stage and late-stage tumor groups, increased mtDNA content was strongly associated with poor survival in the latter, but not in the former, as supported by a previous study that high mtDNA copy number may contribute to the high bioenergetic function of mitochondria and further confer an advantage for malignant behaviors of cancer cells, such as tumor invasion [39].

The article "Variable copy number of mitochondrial DNA (mtDNA) predicts worse prognosis in advanced gastric cancer patients" was published in 2013. Journal: Diagn Pathol.

## Conclusion

In summary, we investigated relative mtDNA content in a large cohort of gastric cancers, and demonstrated that variable mtDNA content was closely associated with lymph node metastasis and higher mortality of the patients with late-stage tumors. Moreover, increased mtDNA content predicts worse survival for the patients with late-stage tumors. Thus, variable mtDNA content may be a valuable biomarker in evaluating poor prognosis of advanced gastric cancer patients.

## Competing interests

The authors declare that they have no competing interests.

## Authors’ contributions

PH conceived and designed the experiments. GZ, YQ and SD performed the experiments. GZ and QY collected the samples and analyzed the data. BS and PH contributed reagents/materials/analysis tools. PH Wrote the paper. All authors are in agreement with the content of the manuscript and this submission.

## References

[B1] JemalABrayFCenterMMFerlayJWardEFormanDGlobal cancer statisticsCA Cancer J Clin20118699010.3322/caac.2010721296855

[B2] BlakelyAMMinerTJSurgical considerations in the treatment of gastric cancerGastroenterol Clin North Am2013833735710.1016/j.gtc.2013.01.01023639644PMC4467541

The article "Variable copy number of mitochondrial DNA (mtDNA) predicts worse prognosis in advanced gastric cancer patients" was published in 2013. Journal: Diagn Pathol.

[B3] TanVPWongBCGastric cancer chemoprevention: the current evidenceGastroenterol Clin North Am2013829931610.1016/j.gtc.2013.02.00123639642

[B4] AllgayerHHeissMMSchildbergFWPrognostic factors in gastric cancerBr J Surg199781651166410.1002/bjs.18008412069448610

[B5] SotoudehKHashemiFMadjdZSadeghipourAMolanaeiSKalantaryEThe clinicopathologic association of c-MET overexpression in Iranian gastric carcinomas; an immunohistochemical study of tissue microarraysDiagn Pathol201285710.1186/1746-1596-7-5722640970PMC3408322

[B6] YamaguchiTFujimoriTTomitaSIchikawaKMitomiHOhnoKShidaYKatoHClinical validation of the gastrointestinal NET grading system: Ki67 index criteria of the WHO 2010 classification is appropriate to predict metastasis or recurrenceDiagn Pathol201386510.1186/1746-1596-8-6523607525PMC3649937

[B7] LiuXXiongHLiJHeYYuanXCorrelation of hK6 expression with tumor recurrence and prognosis in advanced gastric cancerDiagn Pathol201386210.1186/1746-1596-8-6223587030PMC3674969

[B8] ShanLYingJLuNHER2 expression and relevant clinicopathological features in gastric and gastroesophageal junction adenocarcinoma in a Chinese populationDiagn Pathol201387610.1186/1746-1596-8-7623656792PMC3655831

[B9] YasuiWOueNAungPPMatsumuraSShutohMNakayamaHMolecular-pathological prognostic factors of gastric cancer: a reviewGastric Cancer20058869410.1007/s10120-005-0320-015864715

[B10] CorsoGVelhoSParedesJPedrazzaniCMartinsDMilaneziFPascaleVVindigniCPinheiroHLeiteMMarrelliDSousaSCarneiroFOliveiraCRovielloFSerucaROncogenic mutations in gastric cancer with microsatellite instabilityEur J Cancer2011844345110.1016/j.ejca.2010.09.00820937558

[B11] YaoDShiJShiBWangNLiuWZhangGJiMXuLHeNHouPQuantitative assessment of gene methylation and their impact on clinical outcome in gastric cancerClin Chim Acta2012878779410.1016/j.cca.2012.01.01322285775

[B12] QuYDangSHouPGene methylation in gastric cancerClin Chim Acta2013853652366918610.1016/j.cca.2013.05.002

[B13] ShiJYaoDLiuWWangNLvHZhangGJiMXuLHeNShiBHouPHighly frequent PIK3CA amplification is associated with poor prognosis in gastric cancerBMC Cancer201285010.1186/1471-2407-12-5022292935PMC3299648

[B14] ShiJYaoDLiuWWangNLvHHeNShiBHouPJiMFrequent gene amplification predicts poor prognosis in gastric cancerInt J Mol Sci201284714472610.3390/ijms1304471422606006PMC3344242

[B15] YasuiWOueNKuniyasuHItoRTaharaEYokozakiHMolecular diagnosis of gastric cancer: present and futureGastric Cancer2001811312110.1007/PL0001173311760076

[B16] YokozakiHYasuiWTaharaEGenetic and epigenetic changes in stomach cancerInt Rev Cytol2001849951124359710.1016/s0074-7696(01)04003-7

The article "Variable copy number of mitochondrial DNA (mtDNA) predicts worse prognosis in advanced gastric cancer patients" was published in 2013. Journal: Diagn Pathol.

[B17] HatefiYThe mitochondrial electron transport and oxidative phosphorylation systemAnnu Rev Biochem198581015106910.1146/annurev.bi.54.070185.0050552862839

[B18] WallaceDCMitochondria and cancerNat Rev Cancer201286856982300134810.1038/nrc3365PMC4371788

[B19] ShadelGSExpression and maintenance of mitochondrial DNA: new insights into human disease pathologyAm J Pathol200881445145610.2353/ajpath.2008.07116318458094PMC2408405

[B20] ChinneryPFHudsonGMitochondrial geneticsBr Med Bull2013813515910.1093/bmb/ldt01723704099PMC3675899

[B21] CopelandWCWachsmanJTJohnsonFMPentaJSMitochondrial DNA alterations in cancerCancer Invest2002855756910.1081/CNV-12000215512094550

[B22] LanQLimULiuCSWeinsteinSJChanockSBonnerMRVirtamoJAlbanesDRothmanNA prospective study of mitochondrial DNA copy number and risk of non-Hodgkin lymphomaBlood200884247424910.1182/blood-2008-05-15797418711000PMC2582005

[B23] HosgoodHD3rdLiuCSRothmanNWeinsteinSJBonnerMRShenMLimUVirtamoJChengWLAlbanesDLanQMitochondrial DNA copy number and lung cancer risk in a prospective cohort studyCarcinogenesis2010884784910.1093/carcin/bgq04520176654PMC2864414

[B24] LynchSMWeinsteinSJVirtamoJLanQLiuCSChengWLRothmanNAlbanesDStolzenberg-SolomonRZMitochondrial DNA copy number and pancreatic cancer in the alpha-tocopherol beta-arotene cancer prevention studyCancer Prev Res (Phila)201181912191910.1158/1940-6207.CAPR-11-000221859925PMC3208722

[B25] ShenJPlatekMMahasnehAAmbrosoneCBZhaoHMitochondrial copy number and risk of breast cancer: a pilot studyMitochondrion20108626810.1016/j.mito.2009.09.00419788937PMC5040184

[B26] QuFLiuXZhouFYangHBaoGHeXXingJAssociation between mitochondrial DNA content in leukocytes and colorectal cancer risk: a case–control analysisCancer201183148315510.1002/cncr.2590621246538

[B27] XingJChenMWoodCGLinJSpitzMRMaJAmosCIShieldsPGBenowitzNLGuJde AndradeMSwanGEWuXMitochondrial DNA content: its genetic heritability and association with renal cell carcinomaJ Natl Cancer Inst200881104111210.1093/jnci/djn21318664653PMC2720693

[B28] WuCWYinPHHungWYLiAFLiSHChiCWWeiYHLeeHCMitochondrial DNA mutations and mitochondrial DNA depletion in gastric cancerGenes, Chromosomes Cancer20058192810.1002/gcc.2021315892105

[B29] LeeHCYinPHLinJCWuCCChenCYWuCWChiCWTamTNWeiYHMitochondrial genome instability and mtDNA depletion in human cancersAnn N Y Acad Sci2005810912210.1196/annals.1338.01115965052

[B30] LiaoLMBaccarelliAShuXOGaoYTJiBTYangGLiHLHoxhaMDioniLRothmanNZhengWChowWHMitochondrial DNA copy number and risk of gastric cancer: a report from the Shanghai Women’s Health StudyCancer Epidemiol Biomarkers Prev201181944194910.1158/1055-9965.EPI-11-037921784958PMC3169741

[B31] HouPLiuDShanYHuSStudemanKCondourisSWangYTrinkAEl-NaggarAKTalliniGVaskoVXingMGenetic alterations and their relationship in the phosphatidylinositol 3-kinase/Akt pathway in thyroid cancerClin Cancer Res200781161117010.1158/1078-0432.CCR-06-112517317825

The article "Variable copy number of mitochondrial DNA (mtDNA) predicts worse prognosis in advanced gastric cancer patients" was published in 2013. Journal: Diagn Pathol.

[B32] WallaceDCA mitochondrial paradigm of metabolic and degenerative diseases, aging, and cancer: a dawn for evolutionary medicineAnnu Rev Genet2005835940710.1146/annurev.genet.39.110304.09575116285865PMC2821041

[B33] VerschoorMLUngardRHarbottleAJakupciakJPParrRLSinghGMitochondria and cancer: past, present, and futureBiomed Res Int201386123692350975310.1155/2013/612369PMC3581248

[B34] RobinEDWongRMitochondrial DNA molecules and virtual number of mitochondria per cell in mammalian cellsJ Cell Physiol1988850751310.1002/jcp.10413603163170646

[B35] Clay MontierLLDengJJBaiYNumber matters: control of mammalian mitochondrial DNA copy numberJ Genet Genomics2009812513110.1016/S1673-8527(08)60099-519302968PMC4706993

[B36] BurgartLJZhengJShuQStricklerJGShibataDSomatic mitochondrial mutation in gastric cancerAm J Pathol19958110511117573355PMC1871018

[B37] TamuraGNishizukaSMaesawaCSuzukiYIwayaTSakataKEndohYMotoyamaTMutations in mitochondrial control region DNA in gastric tumours of Japanese patientsEur J Cancer1999831631910.1016/S0959-8049(98)00360-810448277

[B38] LinCSChangSCWangLSChouTYHsuWHWuYCWeiYHThe role of mitochondrial DNA alterations in esophageal squamous cell carcinomasJ Thorac Cardiovasc Surg2010818919710.1016/j.jtcvs.2009.04.00719660406

[B39] LinCSLeeHTLeeSYShenYAWangLSChenYJWeiYHHigh mitochondrial DNA copy number and bioenergetic function are associated with tumor invasion of esophageal squamous cell carcinoma cell linesInt J Mol Sci20128112281124610.3390/ijms13091122823109849PMC3472741

